# Innovation of Tin Oxide Ceramic Manufacturing Process Based on WSN and Remote Visualization Technology

**DOI:** 10.1155/2022/4151421

**Published:** 2022-06-15

**Authors:** Junyan Wu, Zhihao Wang

**Affiliations:** ^1^School of Material Science and Engineering, University of Jinan, Jinan, Shandong 250022, China; ^2^School of Material Science and Engineering, Qilu University of Technology (Shandong Academy of Sciences), Jinan, Shandong 250353, China

## Abstract

A wireless sensor network (WSN) collects information from small sensors, processes the information effectively through a built-in computing system, forms a dynamic network topology in a self-organizing method, and sends it to the base station through wireless communication. At the same time, the scale of data generated by high-performance scientific computing has rapidly increased from GB and TB to EB. The traditional scientific vision postprocessing model that initially saved the data and then performed the vision processing became a very time-consuming and troublesome process due to the limitation of disk I/O efficiency, which seriously affected the development of technology, and the accuracy was relatively low. The development of high-performance computer parallel processing technology has promoted parallel visualization, and the expansion of Internet bandwidth has accelerated remote visualization. SnO_2_, or tin oxide, is a kind of N-type semiconductor material with a rutile structure. The crystal structure is stable, the corrosion resistance is good, the melting point is high, the resistance after doping is low, and the sinterability is good. Materials that are sensitive to optics, electrodes, and gases have a wide range of uses. This paper proposes a new data fusion algorithm based on BP neural network and studies the key technologies for the design and implementation of a web-based multiuser remote interactive vision system. In this paper, the effects of ZnO, MnO_2_, Nb_2_O_5_, CuO, and Li_2_CO_3_ doping on the conductivity and bulk density of SnO_2_ semiconductor ceramics were studied by means of ceramic preparation method, using intelligent resistance meter, bulk density tester, X-ray diffractometer, and scanning electron microscope, thus promoting the innovation of tin oxide ceramic preparation process.

## 1. Introduction

The wireless sensor network is a large area of small, cheap, general-purpose battery-supply sensors all over the monitoring area. Nodes can collect surrounding data and information. After comprehensive analysis and processing, it is transmitted to the base station by wireless transmission to form an integrated intelligent information monitoring system outside the area [1]. The development of high-performance computer parallel processing technology has promoted parallel visualization, and the expansion of Internet bandwidth has accelerated remote visualization [2]. When a parallel visualization server is established on a high-performance computer, effective parallel visualization processing can be performed on scientific computing data within time, realizing multiuser remote interactive visualization, which not only greatly improves the visualization efficiency of a large amount of data, but also improves the convenience of visualization tools for high-performance computing users [3]. Integrate scientific calculation process and visualization process, maximize the use of the advantages of high-performance computers, and prevent waste of resources [4–6]. Extracting important information from data quickly and effectively, promoting the interaction between humans and computers, and observing and mining important information in data have become the main subject of large-scale data visualization [7, 8]. Realize the sending of data, which is finally received by the user. The wireless sensor network (WSN), as a new generation of intelligent networks, is developing rapidly. WSN uses sensor nodes to monitor and collect relevant data, integrate and process data information, to perform wireless transmission on the dynamic topology of the self-organizing network, and finally transmit the data results to the sink node [9]. Metal oxide semiconductors such as tin oxide are important gas-sensitive materials, but there is an obvious defect in the porous thick-film tin oxide gas sensors on the market; that is, they require a high operating temperature, which increases their energy consumption on the one hand [10]. On the one hand, it also causes the cross-response of other reducing gases, which reduces the service time of the sensor, so its application range is severely restricted. Room temperature gas sensors made of low-dimensional nanostructured oxide semiconductors have appeared in the laboratory, but they also have some inherent shortcomings that make them difficult to apply to date [11]. In this paper, a catalyst-oxide semiconductor composite form is used to prepare a variety of catalyst-tin oxide composite ceramics, which have a significant response to hydrogen and carbon monoxide at room temperature. These bulk composite ceramics show great application prospects, such as machinery high strength, good preparation consistency, simple process, low cost, and sensitive response [12]. Through a large number of experiments, this research screened out those systems that had obvious response to the target gas at room temperature, and comprehensively characterized the room temperature gas sensitivity of several composite porous ceramics with excellent comprehensive performance, including moisture resistance and time stability, and the formation mechanism was deeply analyzed [13].

## 2. Related Work

The literature adopts a catalyst-oxide semiconductor composite form to prepare a variety of catalysts-tin dioxide composite ceramics, which have a significant response to hydrogen and carbon monoxide at room temperature. These bulk composite ceramics show great application prospects. For example, the mechanical strength is high, the preparation consistency is good, the process is simple, the cost is low, and the response is sensitive [14]. Neither of these two references is a mistake. It is my own fault. This section does refer to 2 references of [13, 15]. And the formation mechanism was deeply analyzed. The literature has developed anode materials with high electrochemical catalyst oxidation activity, excellent performance, and long-term durability, as well as electrochemical reactors with improved electrochemical diffusion control [16]. In order to improve the electrochemical catalytic oxidation activity, the characteristics of the tapered film on the SnO_2_ matrix and the prepared SnO_2_ microporous tube ceramic membrane electrode were studied. In the literature, the tin dioxide microporous tubular ceramic membrane electrode is combined with membrane filtration technology, and a self-designed electrochemical reactor is used to decompose simulated wastewater [17]. According to the requirements of multiuser remote interactive visualization technology for building a parallel visualization server on a high-performance computer, this article focuses on the analysis of the existing remote visualization technology and platform development, design, and implementation of multiple main technologies [18]. Web-based user remote interactive visualization system session uses image transmission. Based on the actual needs of the seminar on the intelligent fitting process, the paper analyzes the literature and existing models, combined with digital dual technology, and proposes a web-based digital workstation dual model that details all levels of the model and the differences and relationships between the models [19]. Based on the workshop and model of the manufacturing process, the detailed model, remote online monitoring, analysis and management of the pipe joint processing workshop are realized. The literature mainly studies the multisource data fusion technology based on related theories and designs and implements the multisource data fusion strategy based on evidence theory. At the same time, it also introduces the transformer fault diagnosis railway transportation system. Finally, an example is selected to verify the function of the system, and good results are achieved [20].

## 3. Wireless Sensors and Remote Visualization Technology

### 3.1. Wireless Sensor

The WSN technology, which is a combination of low-cost small energy-saving sensors capable of short-range communication, has attracted much attention. The node forms a dynamic network topology through self-organization, performs information synthesis and information processing, and sends it to the base station through wireless transmission. In addition, since the location of each sensor is not determined before the design of the wireless sensor network, the node itself does not know the location. First, the WSN node performs data recognition. Then, the processor module will play a role in saving and processing the conversion results. At the same time, the module also receives processing data sent from other nodes. Finally, after the node processing is completed, the wireless communication module sends the result of processing the data to the network monitoring management center. In the whole process, the energy of the node is provided by the energy supply module.

Through the WSN network configured with multiple sensor nodes in the test area, after the dynamic topology of the network is configured in the area, the nodes are dispersed without clearing the nodes in advance, and the surrounding surveillance objects, perception, and collection of large amounts of data information started to be implemented. The node information is integrated with the equipment, and the characteristic value information of the monitoring and fusion data is sent through the route formed on the network. The final result will be sent to the aggregation node, and its information will be sent to the mission management center via the Internet and satellite.  Figure 1 shows the structure of the WSN network.

Task management center is responsible for receiving monitoring function information from the network and can also send instructions to the monitoring area.

Sink node (base station) has powerful processing, storage, and communication functions and sufficient energy.

Sensor network is the main part of the entire wireless sensor network. There are many sensor nodes scattered in high density on the network. These nodes monitor the surrounding environment in real time and send the collected data to the sink node through their own path, or accept the task assigned to the sink node from the task management center. The processor module of each sensor node is a small embedded system used to store and process the data collected by monitoring. In addition, it is usually employed for the use of batteries for energy supply. These functions serve to integrate a large amount of collected data and information and send them to the sink node through wireless communication technology.

The key technologies of WSN mainly include the following.

#### 3.1.1. Network Security Technology

Network security is an important guarantee for the normal operation of the network. If the security of the network is not guaranteed, it is easy for others to steal important confidential information during the sending process.

#### 3.1.2. Time Synchronization Technology

Time synchronization is the work of a wireless sensor network united by many nodes. However, depending on the environment of the node, the requirements of the time synchronization mechanism of each wireless sensor network are also different. Therefore, time synchronization technology is very important for wireless sensor networks.

#### 3.1.3. Node Positioning Technology

In WSN, determining the location information of the node itself and its area is an indispensable step for data collection. Nodes design their own positioning modes according to various network requirements, which are affected by communication interference and other factors, and the energy efficiency used can meet the requirements of self-organization and decentralized computing and other requirements. This is an important topic for current and future research.

#### 3.1.4. Data Fusion

According to the characteristics of WSN, the data information collected by the node from the surrounding monitoring objects contains a lot of redundant information and error information. If the information is sent without processing, the energy of the node will be consumed rapidly, and the life cycle of the network will be shortened. Therefore, after the data information is collected by the node, the sensor network uses this technology to also reduce the bad influence on the sensor node that is vulnerable to failure. Of course, while data fusion technology restrains energy consumption and improves information accuracy, it also has problems such as network delay and increased robustness.

### 3.2. Remote Visualization

The methods used for remote visualization can be divided into the following categories.

Moving the original data. Move the data set from the remote server to the scientific workstation, and process it on the client's high-end visual workstation.

Mobile data sampling. Data sampling is a set of important functions and is part of the original data. Although the amount of data transferred from remote workstations/servers will be reduced, in order to operate and draw these functions, moderate computing power and complex interfaces are required.

Moving the image. The third method is to visualize the data on the remote cluster and stream the image to the scientific workstation. This method requires less bandwidth and little space. The disadvantage is that due to the limited presentation of data available to users, more preprocessing is required, and it cannot be flexibly applied (as shown in Figure 2).

The remote interactive visualization system for high-performance computing data includes the structure shown in the figure. The visual service corresponds to the Java Script background processing of the web client layer. The web service layer of the architecture integrates various visual tools to support remote calls. The following describes the visual conversation application examples.

High-performance remote interactive visualization system generates new image frames based on visual metadata. This interface returns to the wavelet of the web service. And Image Deliver returns the frame of the image. The web server creates new event types based on the event response mechanism. The paint will update the image. The web server obtains the user list of the current visual session and realizes the synchronization of multiple clients.

All conversations between the browser client and the web server are based on requests. The visualization request is issued by the customer, as shown in Figure 3.

### 3.3. Data Principle

This article adopts the energy consumption mode of wireless communication, and the energy consumption is expressed by (1) and (2):

(1) $$\begin{array}{c} E_{Tx}\left(k,d\right)=\left\{\begin{array}{c} E_{elec}*k+E_{fs}*k*d^{2},d<d_{0}\\ E_{elec}*k+E_{mp}*k*d^{4},d\geq d_{0} \end{array}\right.\text{.} \end{array}$$

When node *j* receives the data sent by node I, the energy consumed is as follows:

(2) $$\begin{array}{c} E_{Rx}\left(k\right)=E_{elec}*k\text{.} \end{array}$$

The first cluster head selection process of the DHCP comprehensively considers the aggregation degree and energy consumption of nodes. At the network initialization time, all the aggregation degrees of the Pd sensor nodes are set to 1, and the data is collected and sent. The first cluster head node in the network is selected as the average aggregation degree, and the weight of the next round is calculated. In the selection of cluster heads, the first cluster head node is selected according to the average degree of aggregation to calculate the threshold for the first cluster head selection in the next round. The selection of the first cluster head adopts the calculation formula of the threshold value given in the following formula:

(3) $$\begin{array}{c} \text{T}\left(n\right)=\left\{\begin{array}{c} \frac{p}{1-p*\left(rmod1/p\right)}\left(w_{1}Pd+w_{2}\frac{E_{remain}}{E_{init}}\right),n\in G\\ 0,n\notin G \end{array}\right.\text{.} \end{array}$$

The energy loss of nodes in the network is mainly concentrated in the fusion part of message sending and receiving and data processing, so the energy threshold ETH can be calculated according to the following formula.

(4) $$\begin{array}{c} E_{th}=N_{collect}\times \left(\left(C_{average}-1\right)\times l\times E_{elec}+C_{average}\times l\times E_{DA}+l\times \left(E_{elec}+E_{fs}d_{0}^{2}\right)+l\times E_{DA}\right)=N_{collect}\times \left(C_{average}\times l\times \left(E_{elec}+E_{DA}\right)+l\times E_{DA}\times E_{fs}\times d_{0}^{2}\right)\text{.} \end{array}$$

The DHCP uses intracluster single-hop routing and intercluster multihop routing, and intercluster multihop routing introduces the concept of the second cluster head. The second cluster head is only responsible for sending data packets gathered by the first adjacent cluster head. The goal is to find the best way to reduce the energy consumption of data transmission between clusters. In the process of intercluster routing, the first cluster head of each cluster will select the second cluster head of the cluster that sends the packet. Therefore, after selecting the second cluster head of each cluster, the first cluster head of each cluster must be saved. As shown in Table 1, the information table of the second cluster head of adjacent clusters, the second cluster head of each cluster must also establish a routing information table between the next hop clusters of packets forwarded to other clusters. As shown in Table 2, the second cluster head only needs to save the information of the adjacent second cluster head, and then an appropriate route can be selected. To update the cluster information dynamically, the information table must be rebuilt in each cycle. Tables 1 and 2 are reproduced from Yan and Shi [21].

The setting of the simulation experiment is as follows: randomly configure 100 sensor nodes within a monitoring range of 100 × 100 meters. The main simulation parameters used in the routing protocol are shown in Table 3.

Extract the layer information in the image from the generated two-dimensional image and transfer function. The layers are mainly extracted based on the transparency of each layer in the image and the relevant restriction information of user operations. The main idea is that according to the sample pixels of each layer of the image, the pixels decay exponentially along the line of sight; namely,

(5) $$\begin{array}{c} \text{C}=\overset{D}{\underset{0}{\int }}c\left(s\right)e^{-\overset{D}{\underset{8}{\int }}t\left(t\right)dt}ds\text{.} \end{array}$$

*C*(*s*) represents the reflected light along the line of sight and the incident light of the light source in the sample *S*; then,

(6) $$\begin{array}{c} \text{C}=\overset{L}{\underset{i=1}{\sum }}A_{i}C_{i}\overset{i-1}{\underset{k=1}{\prod }}\left(1-A_{k}\right)\text{.} \end{array}$$

Assuming that the layers of each image are of the same material, the calculation formula for the light of each pixel of the input image is as follows:

(7) $$\begin{array}{c} \text{C}=\overset{L}{\underset{i=1}{\sum }}A_{i}C_{i}\overset{i-1}{\underset{k=1}{\prod }}\left(1-A_{k}\right)\text{.} \end{array}$$

Given a set containing *m* images, it is expressed as follows:

(8) $$\begin{array}{c} \hat{C}=\left\{C_{1},\ldots ,C_{m}\right\}\text{.} \end{array}$$

It represents a collection of *n* layer material colors as follows:

(9) $$\begin{array}{c} \hat{c}=\left\{c_{1},\ldots ,c_{n}\right\}\text{.} \end{array}$$

According to Bayes' inference, the reduction value of each layer of *N* is restored, and that combination becomes as follows:

(10) $$\begin{array}{c} \hat{A}=\left\{A_{1},\ldots ,A_{n}\right\}\text{.} \end{array}$$

According to the Bayesian framework, the *α* reduction value of a layer is the maximum value of the total log likelihood, and the formula is as follows:

(11) $$\begin{array}{c} \text{argmaxP}{\left(\hat{A}|\hat{C,}\hat{c}\right)}_{\hat{A}}=\frac{\text{argmaxP}{\left(\hat{A}|\hat{C,}\hat{c}\right)}_{\hat{A}}\prod_{i=1}^{m}P\left(A_{i}\right)}{\prod_{j=1}^{m}P\left(C_{j}\right)}=\text{argmax}{\left(\text{L}\left(\hat{C,}\hat{c}|\hat{A}\right)+\overset{n}{\underset{i=1}{\sum }}L\left(A_{i}\right)\right)}_{\hat{A}}\text{,} \end{array}$$

(12) $$\begin{array}{c} \text{L}\left(\hat{C,}\hat{c}|\hat{A}\right)=\overset{m}{\underset{j=1}{\sum }}\left(\overset{n}{\underset{i=1}{\sum }}A_{i}c_{i}\overset{i-1}{\underset{k=1}{\prod }}\left(1-A_{k}\right)\right)-C_{j}^{2}/2\sigma_{c_{j}}^{2}\sigma c_{j}\text{.} \end{array}$$

It is assumed that adjacent pixels of the same color should have the same *α* value. The main model is based on the spatial continuity of the maximum similarity theory, which is mainly reflected in the square dispersion of pixels and neighboring pixels.

(13) $$\begin{array}{c} \underset{y\epsilon N\left(x\right)}{\sum }W\left(x,y\right){\left(A\left(x-y\right)-A\left(x\right)\right)}^{2}\text{.} \end{array}$$

Here, *N*(*x*) represents the nearby set of *x*, and *W*(*x*, *y*) is mainly a weighted value for avoiding the generation of the cross section boundary of the fault. This is a function of the gradient between adjacent points, as shown below:

(14) $$\begin{array}{c} \text{w}\left(x,y\right)=\text{exp}\left(-\frac{{\left(g{\left(x,y\right)}^{T}\left(x,y\right)\right)}^{2}}{{\left(x,y\right)}^{T}\left(x,y\right)}\right)\text{.} \end{array}$$

We define image quality as follows:

(15) $$\begin{array}{c} f:\text{V}⟶\left\{quality,resolution\right\},V\in \left(0,100\right)\text{.} \end{array}$$

During initialization, the ideal image size ifs of the calculator under the current network bandwidth and theoretical frame rate fps is

(16) $$\begin{array}{c} f:\left\{bw,fps,vs\right\}⟶ifs\text{.} \end{array}$$

The image quality is obtained according to the ratio, and subsequent images are compressed according to the image quality. That is,

(17) $$\begin{array}{c} f:\left\{ifs,cids_{i-1}\right\}⟶diff_{i} \end{array}$$

according to

(18) $$\begin{array}{c} f:\left\{diff_{i}\right\}⟶V_{i}\left\{\begin{array}{c} V_{i-1}+1,diff_{i}<1\\ V_{i-1},diff_{i}=1\\ V_{i-1}-1,diff_{i}>1 \end{array}\right.\text{.} \end{array}$$

## 4. Research on the Innovation of Tin Oxide Ceramic Manufacturing Process Based on Related Technologies

### 4.1. The Main Mechanism Model of Tin Oxide Ceramic Production

The conductivity of a semiconductor on a macroscopic scale looks very large. The conductivity *σ* is determined by the carrier concentration *N* and the carrier mobility *μ*:

(19) $$\begin{array}{c} \sigma =\text{qn}\mu \text{.} \end{array}$$

For conductors, the carrier mobility is mainly affected by the scattering caused by impurities, phonons, photons, etc., while in semiconductors, the scattering caused by the grain boundary barrier is the dominant effect on the carrier mobility. Semiconductors without impurities and lattice defects are called true semiconductors (silicon, germanium, etc.). In this kind of semiconductors, the carrier concentration *N* and the energy gap *E*_*g*_ satisfy the following relationship:

(20) $$\begin{array}{c} \text{n}=n_{0}e^{-\frac{E_{g}}{2kT}}\text{.} \end{array}$$

Oxygen molecules in the form of gas *o*2(*gas*) first form adsorbed (physical) oxygen molecules *o*2(*ads*) when they come into contact with the surface of sensitive materials through physical adsorption:

(21) $$\begin{array}{c} O_{2\left(gas\right)}⟶O_{2\left(ads\right)}\text{.} \end{array}$$

The carriers in *N*-type semiconductor oxides are almost all electrons. Because the adsorbed state (physical) oxygen molecules have a strong affinity for electrons, they have greater escape power than semiconductors, making it easier to take out electrons from the semiconductor surface to form a chemical adsorbed into the ionic state of oxygen molecules:

(22) $$\begin{array}{c} O_{2\left(ads\right)}+e^{-}⟶O_{2\left(ads\right)}^{-}\text{.} \end{array}$$

Ionic oxygen molecules will further seize electrons to form oxygen ions, and the electronegativity is further improved:

(23) $$\begin{array}{c} O_{2\left(ads\right)}^{-}+e^{-}⟶2O_{\left(ads\right)}^{-}\text{.} \end{array}$$

The CO molecules in the surrounding environment will first be adsorbed on the surface of sensitive materials and, under certain conditions, combine with oxygen ions to form CO_2_ molecules that are adsorbed on the surface of the material or separated from the material (as shown in Figure 4).

In contact with the reducing *R* gas in the environment, the following two processes will occur:

(1) The reducing *R*(*gas*) is in contact with the oxide semiconductor and exists on the surface of the oxide semiconductor by physical adsorption *R*(*ads*).
  (24) $$\begin{array}{c} {\text{R}}_{\left(gas\right)}⟶R_{\left(ads\right)}\text{.} \end{array}$$
(2) Due to the diffusion movement, the adsorbed gas (*ads*) on the surface of the material will eventually contact with oxygen ions, and then the two react to form oxide RO, and the generated electrons are sent back to the depletion layer on the surface of the oxide semiconductor as charge carriers.
  (25) $$\begin{array}{c} {\text{R}}_{\left(gas\right)}+O_{\left(ads\right)}^{-}⟶\text{RO}+e^{-}\text{.} \end{array}$$

### 4.2. Tin Oxide Ceramic Materials

In this experiment, the traditional solid-phase ceramic preparation process was used to prepare tin dioxide semiconductor ceramics, as shown in Table 4.

The equipment and instruments used in this experiment are shown in Table 5.

In addition to the instruments or equipment in Table 5, glass rods, crucibles, vernier calipers, etc. are also used.

### 4.3. Manufacturing Process of Tin Oxide Ceramics

The manufacturing technology of tin oxide ceramics is based on the experiment of sintering temperature above 1400°C and sintering at a temperature of 1050°C; the purpose of the sintering process and pre-sintering is to remove impurities in the sample, make some of the pores and samples more delicate, and prevent high temperature defects caused during sintering (surface cracks, etc.). Moreover, pre-sintering can transfer some energy to the sample particles, and the sample will become larger after final sintering. The mass fraction of the PVA solution added during the dry pressing process was 8%. Excessive addition will slow down the discharge process of the binder and affect the density of the ceramic, and excessive addition will make it difficult to form and cause the edges of the sample to be scattered. This paper studies the difference in the effect of molding pressure on the bulk density of tin oxide ceramics.  Figure 5 shows the relationship between molding pressure and bulk density. In the photo before 25 MPa, if the pressure increases, the density of the sample will become higher. After 25 MPa, the density change caused by the pressure increase is not large, and the sample is easy to heat when the mold is released. Therefore, this experiment uses a pressure of 25 MPa. The sintering temperature method is within 100°C, and the heating rate is 50°C /h. When the temperature is 100 °C ~ 500°C, the heating rate is 100°C /h; and when the temperature is 500°C to the final target, the heating rate is 200°C /h.

In recent years, the research on the doping modification of tin dioxide has also achieved some results, by doping various rare earth oxides to improve the sinterability and conductivity. For example, doping Mn, Cu, Fe, and Zn improves sinterability and crystal structure, so as to achieve the purpose of increasing density. It can also be doped with Bi, Nb, *W*, *V*, etc. to increase the carrier concentration and improve conductivity. According to some literature analysis and some experiments, SnO_2_ doped with 0.5wt.% La_2_O_3_ has better sintering characteristics. The raw materials can be fully mixed and crushed, and finally passed through a 40 mesh sieve and burned in a high-temperature furnace heated at 1050°C for 2 hours. In this process, the discharge rate of the adhesive is low, and it is heated to 500°C and kept for 2 hours. Then, in order to close the furnace door and sinter with the furnace for cooling, the raw materials were heated at 1400°C, 1430°C, 1450°C, and 1470°C, respectively, for 8 hours. Next, clean the sintered wafer, test the volume density and resistivity, and analyze the physical phase and microstructure. The production process is shown in Figure 6.

## 5. Conclusion

According to the shortcomings of the existing WSN network layer aggregation routing protocol, we propose the dual cluster clustering group protocol DHCP based on the aggregation model. The protocol improves the degree of node aggregation, remaining energy, and nonspatial location to balance energy consumption and improve network performance.

In the case of multiuser remote sensing, the characteristics of the design and implementation of shared sessions based on multiuser collaboration agencies are the constraints from session management to integrated management of visual sessions, using server push technology to apply visual real-time synchronization. Create high-performance computing field searches among multiple users. By adjusting the visualization parameters, you can create data online through a browser and share the visualization results of HPC data.

Not only does the noble metal catalyst-tin dioxide composite porous ceramic have excellent room temperature gas sensitivity, but this performance can also be stored for a long period of time under natural conditions; that is, it has certain antiaging properties. For palladium-tin dioxide composite nano-ceramics, even after half a year of aging, there is still a strong response to carbon monoxide at room temperature, but the response speed and recovery speed are reduced, and it is still capable of detecting low-concentration carbon monoxide ability.

## Figures and Tables

**Figure 1:** Sensor network structure.

**Figure 2:** Implementation method of remote visualization system.

**Figure 3:** Communication mode of remote interactive visualization system.

**Figure 4:** CO reaction process on the surface of N-type semiconductor gas sensor.

**Figure 5:** Density after sintering of samples formed under different pressures.

**Figure 6:** Preparation process of tin dioxide semiconductor ceramics.

**Table 1:** The information table of the adjacent second cluster head selected in the first cluster head.

Logo	Significance
ID	Number of adjacent second cluster head nodes

SRE	The remaining energy of the adjacent second cluster head node

dsCH	The distance from the first cluster head node to the adjacent second cluster head node

**Table 2:** The second cluster head information table.

Logo	Significance
ID	Number of adjacent second cluster head nodes

SRE	The remaining energy of the adjacent second cluster head node

dsCH	The distance from the second adjacent cluster head to the second cluster head of the current cluster

**Table 3:** Simulation parameter table.

Parameter	Value
Test area	(0, 0)∼(100, 100) m
Total number of nodes	100
Base station node distance	（50, 150）
The first cluster head node ratio	0.07
Node initial energy	2 J
Data transmission/reception energy consumption	50 nJ/bit
Idle channel mode parameters	10 pJ/bit/m^2^
Multipath channel mode parameters	0.0013 pJ/bit/m^2^
Node data fusion parameters	50 nJ/bit
Packet length	500 bit
d0	87 m
*W*1	0.4∼0.8
*W*2	0.2∼0.6

**Table 4:** Raw materials used in the experiment.

Name	Chemical formula	Purity	Manufacturer
Tin dioxide powder	SnO_2_	Greater than 99.5%	Yueping Scientific Instrument Co., Ltd.
Antimony trioxide	Sb_2_O_3_	Greater than 99.0%	Yueping Scientific Instrument Co., Ltd.
Niobium pentoxide	Nb_2_O_5_	Greater than 98.0%	Yueping Scientific Instrument Co., Ltd.
Zinc oxide	ZnO	Greater than 97.0%	Yueping Scientific Instrument Co., Ltd.
Lithium carbonate	Li_2_CO_3_	Greater than 98.0%	Yueping Scientific Instrument Co., Ltd.
Copper oxide	CuO	Greater than 99.99%	Yueping Scientific Instrument Co., Ltd.

**Table 5:** Experimental equipment and instruments.

Equipment and instrument name	Model	Manufacturer
Silicon carbide rod high temperature sintering furnace	SX2-6-13	Y City Qianjin Furnace Equipment Co., Ltd.
Silicon molybdenum rod high temperature sintering furnace	SX-77-17	Caixing high temperature component electric furnace factory
X-ray diffractometer	D/Max2500PC	Japanese Science
Scanning electron microscope	JXA-840A	JOEL Corporation of Japan
Constant temperature water bath		Saifu Experimental Instrument Factory

## Data Availability

The data used to support the findings of this study are available from the corresponding author upon request.
